RETRACTED

# microRNA -140-5p inhibits colorectal cancer invasion and metastasis by targeting ADAMTS5 and IGFBP5

**DOI:** 10.1186/s13287-016-0438-5

**Published:** 2016-12-01

**Authors:** Lihui Yu, Ying Lu, Xiaocui Han, Wenyue Zhao, Jiazhi Li, Jun Mao, Bo Wang, Jie Shen, Shujun Fan, Lu Wang, Mei Wang, Lianhong Li, Jianwu Tang, Bo Song

**Affiliations:** 1 Department of Pathology, Dalian Medical University, Dalian, 116044 People’s Republic of China; 2 Teaching Laboratory of Morphology, Dalian Medical University, No. 9 West Section, Lvshun South Road, Dalian, 116044 People’s Republic of China; 3 Key Laboratory of Tumor Stem Cell Research of Liaoning Province, Dalian Medical University, Dalian, 116044 People’s Republic of China; 4 Key Laboratory of Tumor Metastasis Research of Liaoning Province, Dalian Medical University, Dalian, 116044 People’s Republic of China

**Keywords:** Colorectal cancer, microRNA-140-5p, ADAMTS5, IGFBP5, Invasion, Metastasis

## Abstract

**Background:**

Colorectal cancer (CRC) is one of the most common malignancies in the world. microRNA-140-5p (miR-140) has been shown to be involved in cartilage development and osteoarthritis (OA) pathogenesis. Some contradictions still exist concerning the role of miR-140 in tumor progression and metastasis, and the underlying mechanism is uncertain.

**Methods:**

Immunohistochemistry was performed to determine the expressions of ADAMTS5 and IGFBP5 in CRC tissues. Human CRC cell lines HCT116 and RKO were transfected with miR-140 mimic, inhibitor, or small interfering RNA (siRNA) against ADAMTS5 or IGFBP5, respectively, using oligofectamine or lipofectamine 2000. Scratch-wound assay and transwell migration and invasion assays were used to evaluate the effects of miR-140 on the capabilities of migration and invasion. The levels of miR-140 and ADAMTS5 and IGFBP5 mRNA were measured by quantitative real-time polymerase chain reaction (qRT-PCR). Western blot was performed to examine the expression of ADAMTS5 and IGFBP5 proteins.

**Results:**

miR-140 was significantly reduced, whereas ADAMTS5 and IGFBP5 were upregulated, in the human CRC tissues compared to the corresponding normal colorectal mucosa. miR-140 downregulation and ADAMTS5 or IGFBP5 overexpression were associated with the advanced TNM stage and distant metastasis of CRC. There was a reverse correlation between miR-140 levels and ADAMTS5 and IGFBP5 expression in CRC tissues. ADAMTS5 and IGFBP5 were downregulated by miR-140 at both the protein and mRNA levels in the CRC cell lines. The gain-of- and loss-of-function studies showed that miR-140 inhibited CRC cell migratory and invasive capacities at least partially via downregulating the expression of ADAMTS5 and IGFBP5.

RETRACTED

**Conclusions:**

These findings suggest that miR-140 suppresses CRC progression and metastasis, possibly through downregulating ADAMTS5 and IGFBP5. miR-140 might be a potential therapeutic candidate for the treatment of CRC.

## Background

Colorectal cancer (CRC) is one of the most common malignancies and the second most common cause of cancer deaths worldwide [1, 2]. Surgery with or without adjuvant radiation and chemotherapy treatments based on tumor stages have been recommended according to current guidelines. However, there are still patients with early surgery suffering from metastases, especially liver metastases, which can finally result in death [3]. Like other solid cancers, the development of CRC is a multistep progression involving the activation of oncogenes and inactivation of tumor suppressor genes, which will affect all aspects of tumorigenicity of CRC, such as cell proliferation, apoptosis, invasion, and metastasis [4]. Because of the disease complexity, the specific molecular genetic and epigenetic alterations of CRC remain largely unknown.

MicroRNAs (miRNAs) are small (19–25 nucleotides), noncoding, regulatory RNAs that can negatively regulate gene expression by complementary base pairing with the 3′-untranslated region (UTR) of target messenger RNAs (mRNAs), leading to their degradation or repression of mRNA translation [5, 6]. Abnormal expression of miRNAs is suggested to be associated with various human disorders, including cancer, indicating that they play a critical role in the molecular mechanism of cancer pathogenesis and progression [7].

The gene encoding microRNA-140-5p (miR-140) is located in chromosome 16. It was first found as a cartilage-specific expression microRNA. Wienholds et al. [8] and Tuddenham et al. [9] reported that miR-140 was specifically expressed in cartilage tissues of zebrafish and mouse embryos, and later its downregulation was shown to play a critical role in the pathogenesis of osteoarthritis (OA) [10–12]. Importantly, several recent studies have revealed the functions of miR-140 in tumorigenesis. The results from our group showed that ectopic expression of miR-140 in human osteosarcoma and CRC cells can induce cell cycle arrest and inhibit cell proliferation, in part through the suppression of histone deacetylase 4 (HDAC4) [13]. In hepatocellular carcinoma (HCC), miR-140 was found to target TGFBRI and FGF9, and its overexpression could suppress HCC growth and metastasis [14]. In non-small cell lung cancer (NSCLC), miR-140 can target IGF1R and monocyte to macrophage differentiation-associated (MMD) to inhibit tumor growth and metastasis [15]. miR-140 inhibited esophageal cancer cell invasion by targeting slug and the subsequent epithelial-mesenchymal transition (EMT) process [16]. Additionally, several studies indicated that downregulation of miR-140 can promote cancer stem cell (CSC) formation in breast cancer and CRC [17–21]. However, some contradictions still exist concerning the role of miR-140 in tumor progression. Malzkorn et al. [22] reported that miR-140 is one of the increased microRNA candidates in glioma progression from grade II to grade IV. Güllü et al. [23] also found that miR-140 is overexpressed in the invasive ductal breast cancer tissues and lymph node-positive samples. Based on the above studies, we intend to investigate the impact and mechanism of miR-140 on CRC progression.

RETRACTED

A disintegrin and metalloproteinase with thrombospondin motifs (ADAMTS) family is a type of newly discovered, zinc-dependent secreted proteinase consisting of 19 members that share the metalloproteinase domain with matrix metalloproteinases (MMPs) [24]. Among ADAMTSs, ADAMTS5 (aggrecanase-2) is well known for its importance in cartilage destruction [24]. Recently, increasing evidence suggests that ADAMTS5 is involved in cancer development and progression. Nakada et al. [25] reported that ADAMTS5 is upregulated in human glioblastoma compared to the normal brain tissues and its overexpression can enhance the invasive capacity of glioblastoma cells through matrigel which contains brevican, a substrate for ADAMTS5. Another study showed that higher mRNA expression of ADAMTS5 is found in the metastatic foci of head and neck cancer as compared to their corresponding primary tumors as well as normal tissues [26]. Filou et al. [27] reported that ADAMTS5 is the main type of aggrecanase expressed in the laryngeal squamous cell carcinoma (LSCC) and presents a stage-related increase. A more recent study reported that miR-144/451 inhibits breast cancer and head and neck squamous cell carcinoma (HNSCC) metastasis by targeting ADAMTS5 and ADAM10, and the overexpression of these two proteins being significantly associated with lymph node metastasis and pathological grade [28].

Insulin-like growth factor (IGF)-binding proteins (IGFBPs) are important regulators of the IGF signaling pathway which consists of six members [29]. IGFBP5, the most conserved member of the IGFBPs in all vertebrates, has been found to play a role not only in the physical processes, such as cell growth, death, and motility, but also in the pathologic processes such as cancer development and metastasis [30]. IGFBP5 promotes prostate cancer growth in vitro and in vivo [31–33]. The plasma levels of IGFBP5 are 1.5-fold higher in breast cancer-bearing mice than in nontumor-bearing mice and are positively correlated with the tumor size [34]. In a rat colon cancer model, IGFBP5 is among the most upregulated gene by microarray gene expression analysis [35]. Hao et al. [36] reported that the expression of IGFBP5 is increased in breast cancers with axillary lymph node involvement and lymph node metastatic tissues compared with primary breast cancer samples. Wang et al. [37] also found that IGFBP5 is more highly expressed in T1 invasive breast cancer than in normal breast epithelium. Moreover, T1N1 breast cancers are more likely to have moderate and strong positive staining for IGFBP5 than T1N0 cancers.

RETRACTED

These data suggest that ADAMTS5 and IGFBP5 may promote the tumorigenesis and cancer progression. Very interestingly, Miyaki et al. [10] and Tardif et al. [38] have experimentally confirmed that ADAMTS5 and IGFBP5 are the direct targets of miR-140 in HEK293T cells and human OA chondrocytes, respectively. Our previous study has shown that miR-140 inhibits human osteosarcoma and CRC cell growth and is also involved in the chemoresistance to methotrexate and 5-fluorouracil (5-FU) [13]. In the current study, we investigated the suppressive role of miR-140 in CRC progression and the correlation with downregulating ADAMTS5 and IGFBP5.

## Methods

### Cell culture and reagents

The human CRC cell lines, HCT116 and RKO, were purchased from the Cell Bank of the Chinese Academy of Sciences, Shanghai, China. HCT116 cells were maintained in McCoy’s 5A medium (Gibco) and RKO cells were cultured in MEM medium (Gibco) containing 10% fetal bovine serum (FBS; Gibco) in a 5% CO_2_ container at 37 °C.

### Clinical specimens

Sixty CRC patients admitted to the First Affiliated Hospital of Dalian Medical University, Dalian, China, were enrolled in this study. The use of human tissue samples was in accordance with relevant guidelines and regulations, and the experimental protocols were approved by the Medical Ethics Committee of the First Affiliated Hospital of Dalian Medical University. All patients have complete clinicopathological data. The adjacent normal colorectal tissue of each patient within at least 5 cm of the tumor margin [39] was also collected as the negative control. All patients provided written informed consent prior to participation in this study. The CRC specimens were histologically examined by hematoxylin and eosin (H&E) staining.

### Transfections of the miRNA mimics and siRNAs specific for ADAMTS5 and IGFBP5

HCT116 and RKO cells (3 × 10^5^ per well) were plated in six-well plates and then transfected with 100 nM of either miR-140 mimic or negative miRNA (Invitrogen) after 24 h with oligofectamine (Invitrogen) according to the manufacturer’s protocols, respectively. Small-interfering RNAs (siRNAs) specific for ADAMTS5 or IGFBP5 (siADAMTS5 or siIGFBP5) from Invitrogen were transfected with oligofectamine at a final concentration of 100 nM in Opti-MEM I Reduced Serum Medium (Life Technology) according to the manufacturer’s instructions. The transfected cells were harvested for RNA isolation and protein extraction at 24 h and 48 h after transfection, respectively.

RETRACTED

### miR-140 knockdown

To knock down the endogenous miR-140, HCT116 and RKO cells were transfected with 100 nM of scrambled miRNA inhibitor or miR-140 inhibitor by lipofectamine 2000 (Invitrogen) in six-well plates (3 × 10^5^ cells/well), respectively. The miRNA inhibitors were purchased from Invitrogen. Co-transfections of miR-140 inhibitor and siADAMTS5 or siIGFBP5 were the negative control. The transfected cells were harvested for protein extraction at 72 h post-transfection.

### Scratch-wound assay

A scratch-wound assay was performed to evaluate the effect of miR-140 on CRC cell migration. The CRC cells (3 × 10^5^ cells/well) in six-well plates were transfected with miRNAs, miRNA inhibitors, or siRNAs and cultured until reaching confluence. A 10 μl pipette tip was used to scrape the monolayer cells for generating a scratch wound. The wounded surface was washed with 1 × phosphate-buffered saline (PBS) to remove the cell debris and thereafter cultured in the serum-free medium. At 72 h after scrape, the wound closures were photographed with a BZ-8100 microscope (Keyence, Japan).

### Transwell migration and invasion assays

For the transwell invasion assay, 60 μl of matrigel was diluted with precooled serum-free medium in 1:4 ratios and was added to the bottom of the transwell chamber and incubated for 1 h at 37 °C. The parental and transfected cells were resuspended at the density of 1 × 10^6^ cells/ml after starvation for 24 h, then 200 μl of cell suspension (2 × 10^5^ cells) were seeded into the upper chambers (24-well insert; pore size 8 μm), while medium supplemented with 10% FBS (600 μl) was placed in the lower chamber. After incubation at 37 °C for 24 h, cells on the top side of the inserts were removed gently with a cotton swab. The inserts were then fixed by 4% methanol for 15 min and stained with 0.1% crystal violet for 15 min. The average migratory cells were counted by randomly choosing five fields each time under the microscope. The experiments were repeated three times.

For the transwell migration assay, the remaining protocol was the same as the transwell invasion assay except for the pre-coat of the matrigel in the inserts.

### RNA extraction

Total RNA, including miRNA, were isolated from the CRC cells with or without transfection and fresh frozen CRC tissues using TRIzol reagent (Invitrogen) according to the manufacturer’s instructions.

RETRACTED

For human CRC, formalin-fixed, paraffin-embedded (FFPE) specimens, approximately 0.005 g for each sample, were extracted. These samples were deparaffinized with xylene, hydrated by ethanol, and digested with proteinase K. Total RNA was isolated using the High Pure RNA Paraffin Kit (Roche, Germany) according to the manufacturer’s instructions.

### Quantitative RT-PCR

For quantitative real-time polymerase chain reaction (qRT-PCR) analysis of miRNA, cDNA was synthesized using the TaqMan microRNA Reverse Transcription Kit (Life Technologies). qRT-PCR analysis was performed on an Agilent MX3000P instrument. The primers for miR-140 and endogenous control RNU6B were purchased from Ambion. The gene expression (ΔCT) values of miRNA from each sample were calculated by normalizing to RNU6B, and relative quantitation (RQ) values were plotted.

For qRT-PCR analysis of mRNA expression, cDNA was synthesized using the PrimeScript RT Reagent Kit with gDNA Eraser (TaKaRa, Dalian, China). The qRT-PCR amplification for mRNA was performed with SYBR Premix Ex Taq II (TaKaRa) on an Agilent MX3000P instrument. The gene expression (ΔCT) values of mRNA from each sample were calculated by normalizing to GAPDH, and RQ values were plotted. Primers were used as follows:

- ADAMTS5: (forward) 5′- AACTGGGGGTCCTGGGGGTCCTGG -3′
  - (reverse) 5′- CATTTCTTGCCTCACACTGCTCAT -3′
- IGFBP5: (forward) 5′- GGAGGAGCCGAGAACACTG -3′
  - (reverse) 5′- GCGAAGCCTCCATGTGTC -3
- GAPDH: (forward) 5′-GCACCGTCAAGGCTGAGAAC-3′
  - (reverse) 5′-TGGTGAAGACGCCAGTGGA-3′.

### Protein extraction and Western blot

The parental and transfected cells were washed with prechilled PBS and lysed in 1 × RIPA buffer (Sigma, St. Louis). The protein concentration was measured by the Bradford method with BSA (Sigma) as the standard. Equal amounts of protein extract (50 μg) were denatured with 8–10% SDS-PAGE, transferred to PVDF membranes (Millipore), and blocked with 5% non-fat milk in TBST (0.1 M, pH 7.4). Protein abundance of GAPDH (1:500; Abgent) served as a control for protein loading. Each sample was treated with rabbit polyclonal anti-ADAMTS5 (1:250; Abcam) or mouse monoclonal anti-IGFBP5 (1:250; Abcam) primary antibodies at 4 °C overnight. Membranes were incubated with secondary antibodies, HRP-conjugated rabbit/mouse anti-IgG (LI-COR Biosciences), diluted at 1:16,000 in TBST, for 2 h at room temperature. Protein bands were detected by the Odyssey infrared imaging system (LI-COR Biosciences).

### Immunohistochemistry analysis

CRC and normal colorectal tissues were sectioned into 4-μm thickness slides and were incubated with rabbit polyclonal anti-ADAMTS5 (1:50; Abcam) or mouse monoclonal anti-IGFBP5 (1:100; Abcam) overnight at 4 °C in a humidified container. Detection was determined by a Non-biotin Horseradish Peroxidase Detection System and DAB substrate (Dako).

RETRACTED

All samples were observed by two pathologists. If there was a disagreement, the observers would re-examine and reach a consensus. For scoring expression of antibodies, both the intensity and extent of immunopositivity were considered. The dominant staining intensity in tumors was scored as follows: 0 = negative, 1 = weak, 2 = moderate, and 3 = strong. The extent of positive staining tumor cells was scored as follows: <25% = 1, 25–50% = 2, 51–75% = 3, and >75% = 4. The final score was determined by multiplying the intensity and the extent positivity scores, which yielded a range from 0 to 12. The mean score from each individual was calculated in tumor cells. The positive expression for markers was scored as follows: >1, IGFBP5 and >2, ADAMTS5. The positive expression of ADAMTS5 and IGFBP5 was found mainly on the cytoplasm of cells. They were presented as a brown granular material.

### Statistical analysis

Statistical analysis was performed using the SPSS software, version 11.0. The results were expressed as the mean ± standard deviation. Student’s *t* test was used to determine the significance of two groups. Two matched clinical sample groups were analyzed by paired *t* test and two unpaired groups were analyzed by unpaired *t* test. One-way analysis of variance (ANOVA) followed by a Bonferroni-Dunn test was used to compare more than two groups. The correlation between miR-140 and ADAMTS5 or IGFBP5 expression was calculated using Spearman’s correlation coefficient. The chi-square test was used to assess the associations among the positive staining of ADAMTS5 or IGFBP5 and clinicopathological indices. *P* < 0.05 was considered statistically significant.

## Results

### miR-140 expression is reduced in the CRC specimens, and its downregulation is associated with the tumor stage and metastasis

To determine the role of miR-140 in CRC development and progression, we evaluated the expressions of miR-140 in 60 paired CRC specimens and the corresponding normal colorectal tissues using qRT-PCR analysis. We found that miR-140 expression was significantly decreased in the CRC tissues compared with the normal controls (*P* = 0.037, Fig. 1).

**Fig. 1:** miR-140 is decreased in CRC specimens. The qRT-PCR analysis of miR-140 was performed in 60 paired human CRC and the matched adjacent noncancerous tissues. Expression level of miR-140 was normalized by the internal control RNU6B in each sample. *P < 0.05

All cases were then divided into a miR-140 low-expression group (*n* = 28) and a high-expression group (*n* = 32) using the median value as the cut off. The correlation between miR-140 expression and clinicopathological parameters was shown in Table 1. Our results indicated that miR-140 was negatively correlated with tumor stage (*P* = 0.045) and metastasis (*P* = 0.031). No significance was found for age, gender, or histological differentiation. These findings suggested that miR-140 may play a critical role in CRC development and progression.

RETRACTED

**Table 1:** The relationship between miR-140 expression and clinicopathological parameters in colorectal cancer

Characteristics	No. of cases	miR-140 expression		*P* value
		Low (median ≤0.278)	High (median >0.278)	
Age				0.667
< 60 years	22	10	12	
≥ 60 years	38	18	20	
Gender				0.778
Male	33	16	17	
Female	27	12	15	
Tumor size				0.602
< 5 cm	23	12	11	
≥ 5 cm	37	16	21	
Stage				0.045*
I/II	28	1	27	
III/IV	32	27	5	
Differentiation				0.076
Well/moderate	24	13	11	
Poor	36	15	21	
Metastasis				0.031*
No	31	7	24	
Yes	29	21	8	

*P < 0.05

### ADAMTS5 and IGFBP5 are downregulated by miR-140 in HCT116 and RKO cells

Bioinformatics analysis using the computational programs (microrna.org, targetscan.org, and pictar.mdc-berlin.de) has shown that the 3′-UTR of ADAMTS5 or IGFBP5 mRNA contains the putative binding sites of miR-140 (Fig. 2a). The later studies performed by Miyaki et al. [10] and Tardif et al. [38] have experimentally identified that ADAMTS5 and IGFBP5 are the direct targets of miR-140 in HEK293T cells or human OA chondrocytes. To further confirm that the expressions of ADAMTS5 and IGFBP5 are indeed regulated by miR-140 in CRC cells, we transiently transfected either miR-140 mimic or negative miRNA into HCT116 or RKO cells. The successful transfection of miR-140 was verified by qRT-PCR (Fig. 2b). The expressions of ADAMTS5 and IGFBP5 at both protein and mRNA levels were quantified by Western blot and qRT-PCR, respectively. We found that miR-140 inhibited the protein expressions (Fig. 2c) and decreased the mRNA levels of ADAMTS5 and IGFBP5 (Fig. 2d) in both HCT116 and RKO cells compared to the negative controls. Knockdown of ADAMTS5 and IGFBP5 by siRNAs were used as the positive control. These data indicated that ADAMTS5 and IGFBP5 expressions are regulated by miR-140 at the post-transcriptional level in the CRC cells, and this is consistent with the previous results [10, 38].

**Fig. 2:** ADAMTS5 and IGFBP5 are downregulated by miR-140 in CRC cells. **a** The mRNAs of ADAMTS5 and IGFBP5 contain putative binding sites of miR-140. **b** HCT116 and RKO cells were transfected with miR-140 mimic using oligofectamine. Oligofectamine alone (Control) and negative miRNA (NC) were the negative controls. The relative expression of miR-140 was determined by qRT-PCR after normalization to the internal control, RNU6B. *P < 0.05. **c** Protein expressions of ADAMTS5 and IGFBP5 were analyzed by Western blot. CRC cells transfected with siRNA specific against ADAMTS5 (siADAMTS5) and IGFBP5 (siIGFBP5), respectively, were the positive control. The quantitative results of Western blot were analyzed by Gel-Pro Analyzer 4.0 software, and GAPDH was used as a loading control. *P < 0.05. **d** ADAMTS5 and IGFBP5 mRNA levels were measured by qRT-PCR and GAPDH was used as the internal control. *P < 0.05. **e** HCT116 and RKO cells were transfected with miR-140 inhibitor (Anti-miR-140) using lipofectamine 2000. Lipofectamine 2000 (Control), scrambled miRNA inhibitor (Anti-NC) and co-transfection of miR-140 inhibitor and siRNA against ADAMTS5 (140i + siADAMTS5) or IGFBP5 (140i + siIGFBP5) were the negative controls. ADAMTS5 and IGFBP5 proteins were quantified by Western blot. *P < 0.05

Next, we performed loss-of-function analysis to further confirm the regulation of ADAMTS5 and IGFBP5 by miR-140. The endogenous miR-140 was knocked down with inhibitor in HCT116 and RKO cells using lipofectamine 2000. To more accurately verify the regulation between miR-140 and ADAMTS5 or IGFBP5, we co-transfected miR-140 inhibitor and siRNA against ADAMTS5 or IGFBP5, respectively, into the CRC cells and considered it as a negative control. Meanwhile, lipofectamine 2000 alone and scrambled oligonucleotide of miRNA inhibitor were used as the negative control. We found that endogenous miR-140 knockdown can restore the expression of ADAMTS5 or IGFBP5 when compared to the negative controls using Western blot (Fig. 2e). All these results indicated that ADAMTS5 and IGFBP5 are downregulated by miR-140 in CRC cells.

RETRACTED

### miR-140 inhibits the migratory and invasive capacities of CRC cells

Given the clinical significance of miR-140 in the CRC specimens, we then assessed the impacts of miR-140 on the cell migration and invasion using scratch-wound and transwell chamber assays and determined the underlying mechanism. In order to eliminate the effect of cell proliferation, CRC cells were cultured in the serum-free medium when performing the scratch-wound assay. As Fig. 3a showed, the gap was broader in the miR-140-transfection cells compared with the negative controls both in HCT116 and RKO cells, and the wound closure was also significantly inhibited by silenced ADAMTS5 or IGFBP5. The cell migratory capacity as assessed by transwell migratory assay (without matrigel) showed that miR-140 overexpression significantly decreased migration of the HCT116 cells through the chamber compared with the negative controls (55.2 ± 7.5 vs. 107.2 ± 8.5 or 112.3 ± 6.1, *P* < 0.05; Fig. 3b). Similarly, silenced ADAMTS5 or IGFBP5 also reduced the migratory HCT116 cells compared to the negative controls (50.6 ± 2.3 or 47.9 ± 3.6 vs. 107.2 ± 8.5 or 112.3 ± 6.1, *P* < 0.05; Fig. 3b). Similar results were also obtained in RKO cells (Fig. 3b).

**Fig. 3:** miR-140 suppresses the migratory and invasive potentials of CRC cells. **a**, **b** and **c** CRC cells were first transfected with the miRNA mimics or siRNAs. Cell migratory and invasive potentials were then determined by the scratch-wound assay and transwell chamber assays with or without matrigel. **d**, **e** and **f** Similarly, scratch-wound assay and transwell assays with or without matrigel were used to determine the potential for migration and invasion in the miR-140 knockdown CRC cells. The representative pictures were chosen from three independent experiments. The cell numbers passing through the filter are indicated as mean ± SD. *P < 0.05

Transwell invasion assay (with matrigel) showed that HCT116 cells with miR-140 overexpression penetrating through the membrane were remarkably less than those in the negative control groups (41.7 ± 4.5 vs. 83.2 ± 6.1 or 82.6 ± 7.9, *P* < 0.05; Fig. 3c), while silenced ADAMTS5 (32.9 ± 3.8) or IGFBP5 (35.8 ± 2.6) had a similar effect with miR-140 overexpression (Fig. 3c). The results from RKO cells were consistent with the data from HCT116 cells (Fig. 3c). Together, miR-140 inhibits the capacities of migration and invasion of CRC cells in vitro, possibly through targeting of ADAMTS5 and IGFBP5.

### Knockdown of miR-140 promotes the migratory and invasive capacities of CRC cells

So far we have assessed the significance of miR-140 in the CRC migration and invasion using a gain-in approach. In order to further elucidate the impacts of miR-140, we performed a series of knockdown experiments using miRNA inhibitors in HCT116 and RKO cells. As shown in Fig. 3d and e, antagonizing the endogenous miR-140 enhanced the CRC cell migratory potential compared to the negative controls using scratch-wound and transwell migration assays. Similarly, the cell invasion impact caused by endogenous miR-140 was reversed by knock down assay (Fig. 3f). These results are highly consistent with those obtained from exogenous miR-140 overexpression experiments. Thus, miR-140 impairs the migratory and invasive capacities of CRC cells in vitro, possibly via downregulating ADAMTS5 and IGFBP5.

### ADAMTS5 and IGFBP5 are inversely correlated with the expression of miR-140 and enhance the progression and metastasis of CRC

Previously we confirmed that ADAMTS5 and IGFBP5 were downregulated by miR-140 in the CRC cell lines, and miR-140 expression was decreased in the CRC specimens as compared to the normal colorectal tissues. To further prove the regulatory interaction of miR-140 and ADAMTS5 and IGFBP5, we used qRT-PCR to measure the mRNA levels of ADAMTS5 and IGFBP5 in the same CRC cohort. The expressions of ADAMTS5 and IGFBP5 mRNA were dramatically increased in CRC specimens compared with adjacent normal tissues (Fig. 4a; *P* < 0.05), and the expression patterns were inversely correlated with that of miR-140 (Fig. 4b). These data in the clinical specimens further prove the negative regulatory interaction of miR-140 and ADAMTS5 and IGFBP5 concluded from the in vitro experiments.

RETRACTED

**Fig. 4:** ADAMTS5 and IGFBP5 are inversely correlated with the expression of miR-140 and positively correlated with the tumor stage and metastasis of CRC. **a** qRT-PCR analysis of ADAMTS5 and IGFBP5 expressions in 60 pairs of CRC and adjacent nontumorous tissues. **b** Correlation of ADAMTS5 and IGFBP5 and miR-140 expression was analyzed by Spearman correlation test in CRC tissues. **c** Immunohistochemistry analysis of ADAMTS5 and IGFBP5 expressions in CRC tissues. 1, 2, 5 and 6: magnification × 20; and 3, 4, 7 and 8: magnification × 40; 1, 3, 5 and 7: primary sites of tumor tissue; and 2, 4, 6 and 8: noncancerous region of CRC. Scale bar = 100 μm. The results of immunohistochemistry were evaluated by the staining scores. *P < 0.05

We also performed immunohistochemistry to assess the expressions and clinical significance of ADAMTS5 and IGFBP5 proteins in the CRC cohort. As Fig. 4c showed, the positive percentages of ADAMTS5 and IGFBP5 expressions were 74.33% and 68.33%, respectively, in the primary CRC samples. When compared to the adjacent normal tissues (19.71% or 21.34%), the differences reached significance (both *P* < 0.05). These findings are consistent with the ADAMTS5 and IGFBP5 mRNA expressions, indicating that ADAMTS5 and IGFBP5 overexpression are related to the development of CRC.

Next, we analyzed the relationship of ADAMTS5 and IGFBP5 expression with the clinicopathological characteristics of the CRC patients. The results showed that overexpression of ADAMTS5 and IGFBP5 were positively correlated with the TNM stage and metastasis (all *P* < 0.05; Table 2). No significant correlation was found with the remaining parameters (Table 2). Taken together, these results suggest that the expression of ADAMTS5 and IGFBP5 is positively correlated with the progression and metastasis of CRC.

**Table 2:** Correlation between ADAMTS5 and IGFBP5 expression and clinicopathological characteristics in colorectal cancer

Characteristic	No. of cases	ADAMTS5		*P* value	IGFBP5		*P* value
		(+)	(–)		(+)	(–)	
Age				0.467			0.378
< 60 years	22	14	8		16	6	
≥ 60 years	38	18	20		28	10	
Gender				0.564			0.867
Male	33	18	15		27	6	
Female	27	14	13		17	10	
Tumor size				0.745			0.675
< 5 cm	23	13	10		15	8	
≥ 5 cm	37	19	18		29	8	
Stage				0.041*			0.037*
I/II	28	3	25		4	24	
III/IV	32	29	3		28	4	
Differentiation				0.896			
Well/moderate	24	15	9		18	6	
Poor	36	17	19		26	10	
Metastasis				0.027*			0.021*
No	31	5	26		4	27	
Yes	29	27	2		26	3	

*P < 0.05

RETRACTED

## Discussion

The complications arising from metastasis become the major causes of death from cancer. In this study, we revealed a novel mechanism for the inhibition of miR-140 in the CRC progression through targeting ADAMTS5 and IGFBP5. Our interest in miR-140 was due to our previous study that indicates its effects on CRC cell proliferation and chemoresistance [13]. We reasoned that miR-140 may influence CRC progression and be a key regulator in CRC.

Firstly we observed a dramatic decrease in miR-140 in the CRC samples as compared to the adjacent normal tissues (Fig. 1). This is consistent with the results from our previous study [13] and a recent study [21]. More importantly, miR-140 downregulation was significantly associated with advanced clinical stage and distant metastasis of CRC (Table 1). In accordance with our results, Zhai et al. [21] found a more progressive reduction in miR-140 in the metastatic CRC tissues than in the primary tissues, and patients with high miR-140 expression had a much longer survival time, further supporting the inhibitory effect of miR-140 on the CRC metastasis. miR-140 downregulation has also been verified in other solid cancers including HCC, NSCLC, and esophageal cancer [14–16], and miR-140 is negatively associated with tumor stage and metastasis of HCC and NSCLC [14, 15]. The clinical relevance of miR-140 in these tumor samples indicates that miR-140 might be a critical regulator of cancer progression.

We next confirmed the inhibitory effects of miR-140 on the CRC cell migration and invasion in vitro (Fig. 3). Several studies have shown that miR-140 participates in the tumor invasion and metastasis through targeting TGFBR1, FGF9, IGF1R, MMD, and Slug [14–16]. In the current study, we confirmed that ADAMTS5 and IGFBP5 are downregulated by miR-140 in the CRC cell lines (Fig. 2). The inhibition of CRC cell migration and invasion by miR-140 is achieved possibly due to the suppression of ADAMTS5 or IGFBP5 (Fig. 3). Our clinical observations also showed that miR-140 has inverse correlation with ADAMTS5 or IGFBP5 (Fig. 4). Consistent with this, Güllü et al. [23] reported that, immunohistochemically, IGFBP5-negative breast cancer samples have a significantly increased expression of miR-140. However, their results indicated that miR-140 is dramatically increased in the breast cancer samples [23]. This different role of the same miRNA may depend on the types of cell and tissue, and time point [40]. A similar phenomenon exists in the stem cell proliferation. miR-140 inhibits breast or colorectal CSC survival and cancer invasive phenotype via downregulation of SOX2/9 or Smad2 [17–21], whereas, during embryonic bone development, miR-140 drives chondrocyte cell proliferation [8, 9] by targeting HDAC4 and the subsequent transcription of Runx2 [9]. This realization provides a captivating twist to the study of whole-organism functional genomics [40].

RETRACTED

The role of ADAMTS5 in cancer has recently been investigated. However, little is known about its function in CRC. Kim et al. [41] reported that ADAMTS5 is highly methylated in CRC compared to the adjacent normal mucosa. On the contrary, our results showed that ADAMTS5 overexpression in the CRC specimens is associated with the TNM stage and metastasis (Table 2). Knockdown of ADAMTS5 can inhibit the CRC cell migration and invasion (Fig. 3). It is well known that malignant tumors destroy the surrounding extracellular matrix (ECM) before invading and metastasizing [42]. As a metalloproteinase, ADAMTS5 possibly promotes the CRC invasion and metastasis through breaking down the ECM, but further investigations are still required to help explain the function and underlying mechanism of ADAMTS5 in CRC.

Recent studies have demonstrated that IGFBP5 might be a useful biomarker for cancerous tissue and metastasis [31–37], but it also shows the opposite effects depending on cancer cell type and expression method [30, 43–46]. In colon cancer, a study using the rat model revealed that IGFBP5 is one of the top upregulated genes [35]. In accordance with this, we found that IGFBP5 serves as a cancer promoter based on our findings in the clinical CRC cohort and CRC cell lines (Figs. 3 and 4 and Table 2 ). Cell migration is a key step in the tumor metastasis process. Vitronectin (VN), a major ECM component, facilitates its function in diverse cellular processes such as cell migration and cell attachment through interactions with a number of ligands [47]. IGFBP5 has been confirmed to exert a stimulatory effect on cell migration when forming complexes with IGFI and VN in skin keratinocytes and MCF7 breast cancer cells [48, 49]. Furthermore, Yasuoka et al. [50] suggested that IGFBP5 induces cell migration via MAPK-dependent and IGF-I-independent mechanisms.

## Conclusion

In summary, we experimentally prove that miR-140 inhibits CRC cell migration and invasion upon downregulating ADAMTS5 and IGFBP5. ADAMTS5 and IGFBP5 are overexpressed in the CRC specimens and are inversely correlated with the levels of miR-140. miR-140 downregulation and ADAMTS5 and IGFBP5 overexpression contribute to the TNM stage and metastasis of CRC. miR-140 might be a key regulator in CRC progression and metastasis and a potential therapeutic candidate for the treatment of CRC.

RETRACTED

## Abbreviations

ADAMTS: A disintegrin and metalloproteinase with thrombospondin motifs
CRC: Colorectal cancer
ECM: Extracellular matrix
EMT: Epithelial-mesenchymal transition
FBS: Fetal bovine serum
HCC: Hepatocellular carcinoma
IGFBP: Insulin-like growth factor-binding protein
miR(NA): microRNA
MMD: Monocyte to macrophage differentiation-associated
NSCLC: Non-small cell lung cancer
OA: Osteoarthritis
PBS: Phosphate-buffered saline
qRT-PCR: Quantitative real-time polymerase chain reaction
RQ: Relative quantitation
siRNA: Small interfering RNA
VN: Vitronectin
